The article "A Clinical Data Management System for Diabetes Clinical Trials" was published in 2022. Journal: J Healthc Eng.

# A Clinical Data Management System for Diabetes Clinical Trials

**DOI:** 10.1155/2022/8421529

**Published:** 2022-02-24

**Authors:** Aynaz Nourani, Haleh Ayatollahi, Masoud Solaymani-Dodaran

**Affiliations:** ^1^Department of Health Information Technology, Urmia University of Medical Sciences, Urmia, Iran; ^2^Health Management and Economics Research Center, Health Management Research Institute, Iran University of Medical Sciences, Tehran, Iran; ^3^Department of Health Information Management, School of Health Management and Information Sciences, Iran University of Medical Sciences, Tehran, Iran; ^4^Department of Epidemiology, Iran University of Medical Sciences, Tehran, Iran

## Abstract

**Background:**

The use of novel medications and methods to prevent, diagnose, treat, and manage diabetes requires confirmation of safety and efficacy in a well-designed study prior to widespread adoption. Diabetes clinical trials are the studies that examine these issues. The aim of the present study was to develop a web-based system for data management in diabetes clinical trials.

**Methods:**

The present research was a mixed-methods study conducted in 2019. To identify the required data elements and functions to develop the system, 60 researchers completed a questionnaire. The designed system was evaluated using two methods. The usability of the system was initially evaluated by a group of researchers (*n* = 6) using the think-aloud method, and after system improvement, the system functions were evaluated by other researchers (*n* = 30) using a questionnaire.

**Results:**

The main data elements which were required to develop a case report form included “study data,” “participant's personal data,” and “clinical data.” The functional requirements of the system were “managing the study,” “creating case report forms,” “data management,” “data quality control,” and “data security and confidentiality.” After using the system, researchers rated the system functions at a “good” level (6.3 ± 0.73) on a seven-point Likert scale.

**Conclusion:**

Given the complexity of the data management processes in diabetes clinical trials and the widespread use of information technologies in research, the use of clinical data management systems in diabetes clinical trials seems inevitable. The system developed in the current study can facilitate and improve the process of creating and managing case report forms as well as collecting data in diabetes clinical trials.

## 1. Introduction

Diabetes is one of the most common chronic diseases in the world [1, 2]. The statistics show that 451 million people worldwide were diagnosed with diabetes, and this figure is expected to rise to 693 million by 2045 [3]. The number of patients with diabetes is significantly increasing in different countries. For example, according to the International Diabetes Federation, the prevalence of diabetes in Iran was %8.94 in 2017 and this figure is expected to reach %13.64 by 2045 [4]. Diabetes has several complications and may cause disorders in various body organs, such as eyes, kidneys, nerves, heart, and blood vessels [5]. As a result, diabetes is accompanied by different comorbidities [6].

The article "A Clinical Data Management System for Diabetes Clinical Trials" was published in 2022. Journal: J Healthc Eng.

In addition to comorbidities, there are psychological damages that patients with diabetes and their families experience and these can increase health care costs [7, 8]. Given the economic, social, psychological, and health problems that diabetes imposes on a patient, family, and society, managing patients with diabetes seems to be essential. This may happen by creating innovative and more effective methods for preventing, diagnosing, treating, and managing diabetes, for example, through conducting diabetes research [9].

Among different types of research, clinical trials are the most significant type and are considered as a basis for developing diabetes management guidelines [10]. In fact, no new drugs could be offered, and no progress would be seen in the field of diabetes, without clinical trials [11]. Therefore, a significant part of the clinical trials registered in different countries, such as the USA (2.7%) and Iran (3.1%), has been devoted to diabetes over the past 10 years (2010 to 2020) [12, 13].

Clinical trials of diabetes, like other clinical trials, are intricate and multifaceted studies. Each phase of these studies requires cautious, appropriate, and planned management of clinical data. Clinical data management is the process of collecting and validating clinical trial data with the aim of conversion into an electronic format for performing statistical analysis, answering research questions, and ultimately preserving for future research [14, 15]. In fact, this process enables researchers to make the right conclusions about the efficacy, safety, benefits, and potential risks of the product under a study by collecting and managing data properly, reducing missing data, and increasing data quality [16, 17]. Clinical data management is a complex process and at least includes developing case report forms, annotating forms, creating databases, entering data, validating data, managing data discrepancies, medical coding, data mining, locking databases, documenting data management processes, and maintaining data security [16, 18–20].

A clinical data management system is software that supports the data management process during the clinical trial and reduces errors that may happen during manual data management [21]. However, the lack of such a system in research centers, especially in large and multicenter trials, may result in longer study time, extra cost for managing data manually, replication, and other problems such as uncertainty about data quality and quantity, security threats, and compromising the confidentiality of research data [22–24].

The article "A Clinical Data Management System for Diabetes Clinical Trials" was published in 2022. Journal: J Healthc Eng.

The results of the previous study revealed that the process of clinical trials data management is not performed appropriately in Iran [25]. The research centers mostly use paper-based forms to collect data. Moreover, the application of electronic systems is mainly limited to statistical software for data analysis. This is the same for diabetes clinical trials which constitutes a large part of the clinical trials in the country [25]. Therefore, it seems that designing and implementing a data management system based on the scientific principles of clinical research can improve the quality of data and facilitate the process of data management. Therefore, the aim of the present study was to develop a web-based system for data management in diabetes clinical trials.

## 2. Materials and Methods

The present study was completed in 2019. It was a mixed-methods study which was conducted in three phases. Each phase of the study is described hereinafter.

### 2.1. Phase 1: Identifying Required Data Elements and Functions for Designing the System

To identify required data elements and functions for designing the system, data were collected using different research methods in three steps which are described below.

#### 2.1.1. Literature Review

Initially, the literature related to the clinical trial data management systems and their characteristics was reviewed narratively [23, 26–47]. Databases included Web of Science, Scopus, Science Direct, ProQuest, Ovid Medline, and PubMed. The search was conducted over a period of 10 years from 2007 to 2017 by one of the researchers (AN), and other researchers (HA) and (MSD) contributed to the review process [17, 20]. In addition to the literature review, studies related to the diabetes clinical trials were reviewed to extract necessary data elements and functions for the system [44–47].

#### 2.1.2. Exploratory Qualitative Study

An exploratory qualitative study was conducted in January-February 2019, and clinical trial researchers were interviewed by one of the researchers (AN). In this study, data were collected through in-depth semistructured interviews with 16 researchers in three endocrinology and metabolism research institutes. An interview guide was developed based on the literature review and contained 14 questions about different types of diabetes clinical trials, required data for diabetes clinical trials, data collection and data entry methods, data management tools, data quality and security management methods, data analysis and reporting methods, and data management standards [48].

The article "A Clinical Data Management System for Diabetes Clinical Trials" was published in 2022. Journal: J Healthc Eng.

#### 2.1.3. Survey

To identify the main data elements and functional requirements of the system, a questionnaire was developed based on the results derived from the literature review and the qualitative study, and a survey study was conducted in July-August 2019. The questionnaire included 85 items and 14 sections about the required data elements and functions for developing a clinical data management system for diabetes clinical trials. The data elements included the study data (6 items), participants' data (9 items), clinical data (3 items), diabetes data (4 items), laboratory tests data (5 items), socioeconomic data (3 items), lifestyle data (3 items), medication data (3 items), and medical history data (2 items), and the required functions included five categories of functional requirements for managing the study (15 items), creating case report forms (7 items), data management (12 items), data validation and quality control (6 items), and data security and confidentiality (7 items). The face validity and content validity of the questionnaire were assessed by five researchers who were experts in conducting diabetes clinical trials. They were endocrinologists who had experience in designing and conducting at least five diabetes clinical trials. The reliability of the questionnaire was calculated using the Kuder-Richardson correlation coefficient (KR-20 = 0.88). After confirming the validity and reliability, the questionnaire was distributed among diabetes clinical trial researchers across the country by one of the researchers (AN).

The participants were 125 researchers who were experts in conducting diabetes clinical trials. The participants worked in the endocrinology and metabolism research institutes and diabetes research centers affiliated with 11 medical universities across the country. To increase the response rate, the questionnaire was provided in both paper and electronic formats. The link of the online questionnaires was sent to all diabetes clinical trial researchers (*n* = 125). One of the researchers (AN) also attended in person in three endocrinology and metabolism research institutes in the capital and provided the researchers with a paper-based questionnaire (*n* = 39) to improve the response rate. Data were analyzed using descriptive statistics and a cut-off point of 60% agreement was considered to select the necessary items to be included in the system. It means that if at least 60% of the participants agreed on the necessity of including an item in the system, it was considered in the second phase of the study, namely, system development. This cut-off point was also used in the previous studies [49–51]. It helped to include the most necessary items in the system and prevent storing a large volume of data.

The article "A Clinical Data Management System for Diabetes Clinical Trials" was published in 2022. Journal: J Healthc Eng.

### 2.2. Phase 2: Developing a Clinical Data Management System for Diabetes Clinical Trials

In this phase, a clinical data management system for diabetes clinical trials was designed based on the results derived from phase one by one of the researchers (AN). To develop the system, Rapid Prototyping (RP), Microsoft. NET Framework, web design guidelines, and user interface design guidelines for web applications were used. The system prototype was developed in the visual studio using the ASP.NET programming language, and the SQL-Server database management system was used to store data in the system. An Internet Information Service (IIS) for Windows® was also used to maintain the website available 24 hours a day and allows users to access the system at any time of the day or night. Then, the system was hosted on the server to be used by the researchers.

### 2.3. Phase 3: System Evaluation

The purpose of this phase was to evaluate the clinical data management system for diabetes clinical trials from the researchers' perspectives. Initially, the think-aloud method was used to evaluate the usability of the system. The purposive sampling method was used, and the participants who were experts in diabetes clinical trials and expressed their interests in using the new data management system during the first phase of the study were recruited (*n* = 6). According to the literature, five to eight participants are enough for this type of evaluation study [52]. All participants worked in different endocrinology and metabolism research institutes and diabetes research centers affiliated with three medical universities in Tehran. This phase of the research was conducted in the participants' workplace.

To conduct the think-aloud method, a list of tasks (*n* = 26) that covered the whole aspects of the system prototype was given to the participants by (AN). The participants used the system individually, entered sample data from previously completed clinical trials, and expressed their thoughts while performing the tasks. Their role was defined as a clinical trial manager, as this person had access to all sections of the system. Snagit software was used to monitor the participants' activities on the screen and the time taken to undertake the experiment. Moreover, the participants' voices were recorded and notes were taken. The collected data were transcribed, and a content analysis method was used to analyze data. Finally, the usability issues were identified and fixed. The usability issues were mainly related to the users' difficulties with using the interface of the system. They were recognized when a user could not complete a task successfully or when she/he explained difficulties with finding the right way to complete a task.

The article "A Clinical Data Management System for Diabetes Clinical Trials" was published in 2022. Journal: J Healthc Eng.

Then, users' perspectives about the system functions were investigated. In this phase, a convenience sampling method was used, and the participants were invited to take part in the study. The settings of the study were three endocrinology and metabolism research institutes in Tehran. In total, 30 out of 32 diabetes researchers who were experts in conducting diabetes clinical trials accepted to take part in the study. The system was available for two weeks, and during this period, the participants were asked to use the system. The duration of using the system and the tasks they performed could be observed through the system log file. Moreover, one of the researchers (AN) reminded the participants by phone or in person to use the system. They performed all data management tasks as a clinical trial manager because this role had access to different parts of the system. They were also asked to create a clinical trial in the system and enter the test data, as they were not allowed to use the system for a real clinical trial without a legal approval.

To evaluate users' perspectives about the system functions, a questionnaire was designed based on the main functions of the system. The questionnaire included 17 questions and was developed based on a seven-point Likert scale. Such a scale was used to provide a better and more precise reflection of a respondent's perspective. Finally, the data were analyzed using descriptive statistics.

## 3. Results

In the first phase of the study, the questionnaire was distributed among 125 researchers who worked in the endocrinology and metabolism research institutes and diabetes research centers affiliated with 11 medical universities, and 60 researchers (48%) completed the questionnaire. The participants' characteristics are presented in Table 1.

After data analysis, a number of required data elements and system functions for developing the clinical data management system were selected to be included in the system. These items were selected based on the level of agreement among the respondents (agreement of 60% or more).  Table 2 shows some of the required data elements for developing a clinical data management system for diabetes clinical trials and Table 3 illustrates the functional requirements for data quality control.

The article "A Clinical Data Management System for Diabetes Clinical Trials" was published in 2022. Journal: J Healthc Eng.

In the second phase of the study, the prototype of the system was developed using the ASP.NET programming language. Each user had to register in the system primarily and confirm his/her role. The user could select one of the three roles defined in the system. These roles were clinical trial manager (for those studies that the researcher was defined), data supervisor (for those studies that the clinical trial manager invited a researcher as the data supervisor), or data entry operator (for those studies that the clinical trial manager invited a researcher as the data entry operator).  Figure 1 demonstrates the clinical trial management page.

As shown in Figure 1, a clinical trial manager was able to design the diabetes clinical trial, manage other researchers' roles in the trial, develop a case report form, review patient records, provide statistical reports, and lock the database. In “Clinical Trial Design,” the clinical trial manager was able to define the size of a clinical trial (multicenter/single center), the number of participants, the number of phases, the type of randomizations, etc. The clinical trial manager could use the “Users' Roles” menu to define and invite other researchers including the data supervisors or data entry operators. Case report forms could be developed for different phases of the trial, and the clinical trial manager could use “Audit Trial” to view and print all events which occurred in the system. Furthermore, it was possible to view all the activities associated with clinical data management through the “Documentation of Clinical Data Management Process” option. The clinical trial participants' data were available in “Participants' Records.” Each record contained the case report forms of each participant. “Reports and Statistics” provided statistical information about the participated centers in the trial and the number of researchers and participants in the drug and placebo groups. Using the “Database Lock” option, the clinical trial manager was able to lock the database and prevent any data modifications. Finally, the clinical trial manager could return to his/her profile using the “Return to Profile” icon.

Generally, one of the most important tasks for a clinical trial manager is to define the case report forms at the beginning of the study. The current clinical data management system allows the clinical trial manager to select the required data elements for creating case report forms. Moreover, the manager could create the desired forms for each phase of the clinical trial by using different variables (Figure 2).

In the designed system, data supervisors were allowed to review the recorded data for each patient and report or correct any errors or discrepancies using the “Participants' Records” section. Finally, all records could be extracted into Excel or SPSS files for conducting the final analysis.

The article "A Clinical Data Management System for Diabetes Clinical Trials" was published in 2022. Journal: J Healthc Eng.

In the third phase of the study, the usability and users' perspectives about the system functions were evaluated by using the think-aloud method and a questionnaire, respectively. Six researchers who were experts in diabetes clinical trials participated in the usability evaluation study. Most of the participants were female (*n* = 5, 83.3%), and most of them had a Ph.D. degree in different fields, such as epidemiology (*n* = 2, 33.3%), nutrition (*n* = 2, 33.3%), and health education and promotion (*n* = 1, 16.7%). One of the participants was an endocrinologist (*n* = 1, 16.7%), and half of the participants (*n* = 3, 50.0%) had 9–15 years of work experience. A list of tasks was given to the participants, and they were asked to perform the tasks according to the list, while they expressed their opinions loudly.

The results of the usability evaluation showed that some users encountered an error or were unsuccessful in designing a clinical trial (three users), defining study groups (two users), creating case report forms (four users), designing case report forms by using the defined data elements (one user), returning to the personal profile (four users), and logging out (one user). These issues were mainly related to the user interface design which were fixed and the system was improved.

To evaluate the functions of the system from the users' perspectives, 30 researchers took part in the evaluation study. Nearly half of the participants had a subspecialty degree in endocrinology and metabolic diseases (*n* = 14, 46.7%), and the highest frequency was related to those who had 9–15 years of work experience (*n* = 13, 43.3%). The participants used the clinical data management system for two weeks and completed a questionnaire.  Table 4 shows users' perspectives about the system functions.

As Table 4 shows, the total mean value for the system functions was 6.3 ± 0.73. The highest mean values were related to extracting research data (6.9 ± 0.44), ensuring data quality (6.8 ± 0.57), and displaying participants' records (6.7 ± 0.73). The lowest mean value belonged to providing reports by using the system (5.8 ± 0.94).

## 4. Discussion

Currently, many national and international scientific organizations and associations seek funding and build support for diabetes research to generate new knowledge and provide the patients with better care, diagnosis, and treatment [10]. Diabetes clinical trials are among the main types of research which are primarily conducted to answer questions about the efficacy and safety of new medical products and methods and develop new knowledge to deal with diabetes. Finding appropriate answers for these questions and applying new knowledge depends on the correct and systematic collection and management of data [39]. Generally, data management in clinical trial research is a complex process and can be more complicated by an increase in the number of centers involved in a trial, the number of researchers, and the number of study participants [15]. Manual management of this level of complexity is hardly possible. This emphasizes the importance of using clinical data management systems for facilitating this process, improving data quality, and achieving effective results [53].

The article "A Clinical Data Management System for Diabetes Clinical Trials" was published in 2022. Journal: J Healthc Eng.

In the present study, a clinical data management system was developed for diabetes clinical trials. This system was developed based on the data elements and functions suggested by the literature review and diabetes researchers. It should be noted that most clinical data management systems have four main components. The first component includes a management module for designing clinical trial studies, creating case report forms, adding researchers and research centers, maintaining security, and controlling user access. The second component consists of the graphical user interface for entering study data, and the third component is the validation engine for verifying and validating data entered into the database. The fourth component comprises a reporting module to generate the necessary reports about the data and the study process [54].

In the clinical data management system developed in the present study, all four major components were considered. The required data elements were divided into three groups: “study data,” “participant's personal data,” and “clinical data.” These data elements are the minimum data elements required for creating diabetes case report forms. The functions of the system were divided into five main functions, namely, “managing the study,” “creating case report forms,” “data management,” “data quality control,” and “data security and confidentiality.” The management module of this system helped the clinical trial manager to design a clinical trial, add researchers and research centers, define the role of the users, organize the study groups, randomize participants, and edit the trial protocols. These functions have also been considered in other similar systems [23, 39]. For example, in the OpenClinica system, Negari et al. highlighted the role of the clinical trial management module in planning for data management and paid attention to the formation of the study groups (drug and placebo groups), randomizing of the participants, and inviting researchers [39]. In another study, Muller et al. found that the management module of the clinical trial data management system can be useful in the successful management and administration of clinical trials in accordance with the ethical and legal guidelines of the scientific communities [23]. Similarly, Di Leo et al. stated that a management module in clinical data management systems can help centralized management of the study [54].

The article "A Clinical Data Management System for Diabetes Clinical Trials" was published in 2022. Journal: J Healthc Eng.

As mentioned above, another component of a clinical data management system is the graphical user interface for entering clinical trial data. Therefore, a graphical user interface was designed for managing, entering, and reporting data. The user interface of the system was designed using the web-based ASP.NET programming language, which was used in the design of similar systems in other studies [32, 38]. Although there are different programming languages that can be used to design data management systems [27, 30, 41, 43], the .NET framework appears to have comprehensive libraries for developing web-based systems and makes system development easier [55].

Regarding the third component, i.e., data validation, different aspects of data validation and quality control were taken into account in the developed system, so that the clinical trial manager could define multiple validation rules, such as data reentry, data range checking, and data type checking for each field of data. Similar rules have also been considered in other systems such as OpenClinica and REDCap [39, 56]. However, this function was not considered in the other systems such as Ez-Entry, ObTiMA, and OnWARD, and the rules were defined equally for all fields [34, 41, 42]. Some benefits of defining validation rules are reducing data entry time and increasing the accuracy of the entered data [57]. The fourth component of a clinical data management system is the reporting module. In the present study, the system was able to report at different levels in CSV and SPSS formats. In fact, reporting and extracting data are important aspects of the clinical data management process, by which the study data are provided to the supervisors for reviewing and to the statisticians and data analysts for analyzing [18, 58]. Therefore, it is better to prepare this report readable for statistical software such as SPSS and SAS. Similarly, in the present study and other similar research studies [30, 32, 33], CSV and SPSS files were used to extract and report the data and to facilitate analyzing data processes.

Finally, the developed system was evaluated by clinical trial researchers. In terms of usability, most of the problems were related to the user interface design or users' misunderstandings of the terms used in the interface. Although, in many similar studies, the think-aloud method has not been used to evaluate the system prototype [23, 28, 35, 40], we used this method to solve the usability issues and improve user satisfaction and system acceptance [59–61]. The think-aloud method is a reliable subjective measure of user experience. For domains such as usability evaluation, the data generated by using this method can help to improve the user interface. However, one of the weaknesses of this method is that the participant's behavior during doing tasks does not adequately reflect the high level of cognitive processing [62]. Therefore, different evaluation methods should be used together to be able to judge information systems.

The article "A Clinical Data Management System for Diabetes Clinical Trials" was published in 2022. Journal: J Healthc Eng.

As the diabetes researchers had different specialties such as nutrition, health education and promotion, physiology, and epidemiology, and clinical trials conducted by each specialty could be different in terms of the study aim, type of intervention, and data collection, in the present study, different researchers with various backgrounds were invited to evaluate the system functions. Similarly, in other previous studies, researchers with various specialties, characteristics, and skills were involved in the evaluation research [62–64]. According to the results, the system functions were at a good level from the users' perspectives. The users believed that the system worked better in extracting data, controlling data quality, and displaying participants' records. Similarly, in the study conducted by Lee et al., a questionnaire was used to evaluate the developed system in terms of easy logging in and logging out as well as data retrieval [35]. In another study, Micard et al. investigated the system functions in terms of data storage of multicenter trials and the management of text and image files [37]. In the present study, all functions of the system were evaluated from the researchers' perspectives, and the results revealed that they evaluated the system functions at a good level.

## 5. Limitations of the Study

In the current study, a clinical data management system was developed for diabetes clinical trials. To the best of our knowledge, it was the first time that such a system was developed for managing data in a clinical trial; however, there were some limitations that can be addressed in future studies. For example, in the first phase of the study, a cut-off point was considered to include the most necessary items in the system. Although most of the questionnaire's items were found necessary by the majority of the participants, a limited number of the items were removed, because the total level of agreement for these items was less than 60%, and only the necessary items were included in the system design. As the results of the summative evaluation showed, most of the users evaluated the system functions at a good level. Therefore, we believe that the system met their expectations. However, it can be still improved and customized based on the users' requirements in the future.

The article "A Clinical Data Management System for Diabetes Clinical Trials" was published in 2022. Journal: J Healthc Eng.

There were also some limitations regarding system evaluation. In the current study, a prototype of a clinical data management system was developed; therefore, it was not possible to evaluate it in real clinical trials. However, different evaluation methods were used to determine users' opinions about the usability and system functions. Therefore, using the system in real clinical trials and evaluating it by using other evaluation methods and more users are recommended.

## 6. Conclusions

In the present study, a clinical data management system was developed and evaluated to support the data management process in diabetes clinical trials. In this system, the data elements included study data, participant's personal data, and clinical data, and the system functions covered managing the study, creating case report forms, data management, data quality control, and data security and confidentiality. The results of the evaluation study revealed that the researchers generally evaluated the system functions at a good level. It seems that the developed system can be efficient in practice and facilitates the clinical data management process in endocrinology and metabolism research institutes and diabetes research centers. Furthermore, it can be useful for cooperation between the diabetes research centers located in different geographical areas, as it can support data management processes in multicenter clinical trials. However, further investigations are needed to address the cost-effectiveness of the system and compare the data quality and documentation processes before and after using the system in real clinical trials.[65].

## Figures and Tables

**Figure 1:** Diabetes clinical trial management.

**Figure 2:** Creating a case report form for a diabetes clinical trial.

**Table 1:** The participants' characteristics in the first phase of the study.

Variables		Frequency (%)
Sex	Male	26 (43.3)
	Female	34 (56.7)

Age	26–35	9 (15.0)
	36–45	22 (36.7)
	46–55	20 (33.3)
	56–65	9 (15.0)

Education level	Subspecialist	15 (25.0)
	Specialist	9 (15.0)
	PhD	30 (50.0)
	M.Sc.	6 (10.0)

Field of study	Endocrinology	14 (23.4)
	Nutritional sciences	9 (15.0)
	Epidemiology	7 (11.7)
	Obstetrician	4 (6.7)
	Traditional medicine	4 (6.7)
	Internal medicine	4 (6.7)
	Nursing	4 (6.7)
	Clinical psychology	4 (6.7)
	Physiology	2 (3.2)
	Pregnancy health	2 (3.2)
	Social medicine	2 (3.2)
	Pharmacology	1 (1.7)
	Health education and promotion	1 (1.7)
	Molecular medicine	1 (1.7)
	Clinical pathology	1 (1.7)

Work experience (years)	8–2	22 (36.7)
	15–9	16 (26.7)
	22–16	8 (13.2)
	29–23	7 (11.7)
	37–30	7 (11.75)

The article "A Clinical Data Management System for Diabetes Clinical Trials" was published in 2022. Journal: J Healthc Eng.

**Table 2:** Some of the required data elements for developing a clinical data management system for diabetes clinical trials.

NO	Type of data	Data elements	Necessary(%)	Unnecessary(%)
1	Diabetes data	Type of diabetes	60 (100)	0 (0)
2		Duration of diabetes	60 (100)	0 (0)
3		Number of hypoglycemic attacks (per year)	46 (76.7)	14 (23.3)
4		Diabetes complications	60 (100)	0 (0)

5	Laboratory tests data	Fasting blood sugar	60 (100)	0 (0)
6		Hemoglobin A1C	56 (93.3)	4 (6.7)
7		Insulin level	49 (81.7)	11 (18.3)
8		Cholesterol	54 (90.0)	6 (10.0)
9		Triglyceride	55 (91.7)	5 (8.3)

10	Medication data	Name of the current medications	57 (95.0)	3 (5.0)
11		Dosage of the current medications	51 (85.0)	9 (5.0)
12		Duration of using medications	59 (98.3)	1 (1.7)

13	Medical history data	Family history of diabetes	57 (95.0)	3 (5.0)
14		History of previous diseases	60 (100)	0 (0)

**Table 3:** Functional requirements for data quality control.

NO	Functional requirements	Necessary(%)	Unnecessary(%)
1	Checking double data entry	34 (56.7)	26 (43.3)
2	Displaying required fields	52 (86.7)	8 (13.3)
3	Checking data range	55 (91.7)	5 (8.3)
4	Checking data type	55 (91.7)	5 (8.3)
5	Displaying messages for data entry	57 (95.0)	3 (5.0)
6	Using data validation rules	41 (68.3)	19 (31.7)

**Table 4:** Users' perspectives about the system functions.

#	System functions	Very poor	Poor	Slightly poor	Neutral	Slightly good	good	very good	Mean	SD
1	Creating a new clinical trial	0	0	0	2 (6.7%)	6 (20.0%)	12 (40.0%)	10 (33.3%)	6.0	0.91
2	Designing a clinical trial	0	0	0	2 (6.7%)	8 (26.6%)	12 (40.0%)	8 (26.7%)	5.9	0.90
3	Creating case report forms	0	0	0	1 (3.3%)	7 (23.3%)	16 (53.4%)	6 (20.0%)	5.9	0.76
4	Managing case report forms	0	0	0	1 (3.3%)	6 (20.0%)	14 (46.7%)	9 (30.0%)	6.0	0.81
5	Defining data validation rules	0	0	0	1 (3.3%)	2 (6.7%)	10 (33.0%)	17 (56.0%)	6.4	0.77
6	Defining uses' roles	0	0	0	0	1 (3.3%)	13 (43.3%)	16 (53.4%)	6.5	0.57
7	Managing system users	0	0	0	0	1 (3.3%)	13 (43.3%)	16 (53.4%)	6.5	0.57
8	Managing research centers	0	0	0	0	1 (3.3%)	11 (36.7%)	18 (60.0%)	6.6	0.57
9	Creating participants' records	0	0	0	1 (3.3%)	6 (20.0%)	8 (26.7%)	15 (50.0%)	6.2	0.83
10	Managing participants' records	0	0	0	1 (3.3%)	6 (20.0%)	8 (26.7%)	15 (50.0%)	6.2	0.83
11	Entering participants' data	0	0	0	0	1 (3.3%)	10 (33.3%)	19 (63.4%)	6.6	0.56
12	Displaying participants' records	0	0	0	1 (3.3%)	1 (3.3%)	4 (13.3%)	24 (80.1%)	6.7	0.73
13	Ensuring data security	0	0	0	1 (3.3%)	5 (16.7%)	17 (56.7%)	7 (23.3%)	6.0	0.74
14	Ensuring data quality	0	0	0	0	2 (6.7%)	3 (10.0%)	25 (83.3%)	6.8	0.57
15	Documenting data management process	0	0	0	2 (6.7%)	2 (6.7%)	11 (36.7%)	15 (50.0%)	5.9	0.92
16	Providing research reports	0	0	1 (3.3%)	1 (3.3%)	8 (26.6%)	14 (46.8%)	6 (20.0%)	5.8	0.94
17	Extracting research data	0	0	0	0	1 (3.3%)	2 (6.7%)	27 (90.0%)	6.9	0.44
**Total Mean and SD**									6.3	0.73

The article "A Clinical Data Management System for Diabetes Clinical Trials" was published in 2022. Journal: J Healthc Eng.

## Data Availability

All data generated or analyzed during this study are included in this published article.
